# A Controllable Secure Blockchain-Based Electronic Healthcare Records Sharing Scheme

**DOI:** 10.1155/2022/2058497

**Published:** 2022-03-04

**Authors:** Honglei Li, Xiao Yang, Hongxin Wang, Wujia Wei, Weilian Xue

**Affiliations:** Liaoning Normal University, Dalian 116029, China

## Abstract

The sharing of electronic healthcare records (EHRs) is important to healthcare and medical research. However, institutions are faced with difficulties in privacy protection and efficiently secure data exchange. The main objective of this study is to propose a controllable secure blockchain-based EHRs sharing scheme. For this purpose, blockchain technologies are combined with interplanetary file systems (IPFS) to provide efficient secure EHRs sharing. Firstly, the IPFS-based EHR file system (IEFS) is designed to save and share large-size EHR files among medical institutions. With the high-throughput content-addressed block storage model and appropriate redundant backup of IPFS, IEFS is tamper-resistant and free of a single point of failure. Secondly, the blockchain is used to implement the blockchain-based EHR abstract system (BEAS) to manipulate EHR abstracts access. In BEAS, the EHR file addresses generated by IEFS are encrypted and saved in EHR abstracts for privacy protection. Since EHR abstracts are encrypted by patients' public keys, the sharing of EHR files is under the control of patients. In our experiment, a prototype system is developed to validate the proposed scheme. The experimental results showed that (1) EHRs are securely shared under the control of patients and (2) EHR files are retrieved at an acceptable speed supported by IPFS technology. In this paper, solutions to some important practical issues such as incapacitated patients, encryption key forgetting/missing, and efficient interaction of doctors with EHRs sharing scheme are also seriously discussed.

## 1. Introduction

Electronic healthcare records (EHRs) are generated and stored in hospital information systems (HIS), which are often referred to by doctors for disease diagnosis, treatment evaluation, and clinical research. The extensive use of EHRs effectively improves the efficiency and flexibility of medical services. Especially when combined with cloud storage and mobile applications, it can comprehensively improve the convenience, intelligence, and accuracy of the treatment of public healthcare [1, 2]. For serious or chronic diseases, if doctors visit the previous medical records, they can integrate the previous diagnosis and treatment effect with their expertise. As a result, a more comprehensive and accurate diagnosis of the disease is made and more effective treatment is provided. Meanwhile, for serious infectious diseases, EHRs sharing can also enable medical teams in remote regions to make collaborative judgments on the epidemic situation and improve the efficiency of disposal and the level of public healthcare [3].

At present, digitalization and cloud computing technologies have stimulated the demand for EHRs sharing. Considering the medical records involving personal privacy and security issues, only authorized users can access the relevant medical records. Protecting the privacy of personal medical records is not only a moral responsibility but also a mandatory requirement of the law. The secure sharing of EHRs focuses on two issues: one is to effectively prevent unauthorized entities from access to medical records; the other is to enable patients to track and manage their own medical records to increase the transparency of medical services and avoid doctor-patient conflicts. For some important government officials, business executives, and other special groups, once their EHRs are leaked, it may bring serious consequences.

In current medical service systems, hospitals generate and manage EHRs locally. Taking into account the great value of healthcare data and the competitive relationship between providers of medical equipment, there exist exchange barriers of healthcare data among hospitals or other types of medical institutions. In other words, it is difficult to realize the patient-oriented application of healthcare data. Furthermore, data sharing between medical institutions without supervision and control may expose patients' personal privacy and even cause serious damage to their reputation, property, work, and so on [4]. Even in current medical institutions that partially complete electronic medical records, it is difficult to ensure data security if the data are stored on servers or are directly outsourced to third parties. Moreover, the centralized management of EHRs makes them more vulnerable to centralized attack, malicious tampering, and single point failure. It hints that protecting patient privacy and other sensitive data becomes more difficult [5, 6], which easily causes disputes between doctors and patients [7–9]. As a result, the problems of secure sharing of EHRs not only increase the patients' medical service costs but also affect the effective communication and cooperation between medical institutions.

From the legal point of view, EHRs are typical personal private data, which means individuals enjoy absolute ownership, even if they are stored and managed by hospitals. Therefore, for the implementation of effective and reasonable EHRs sharing, patients require sufficient rights and technical support to know and control the access to their own medical records among hospitals. In this paper, a blockchain-based scheme is proposed to secure healthcare data sharing under the control of patients. The proposed scheme encloses the blockchain technology and the interplanetary file system (IPFS) technology in it. In the scheme, EHRs are stored and managed in IPFS and accessed according to the encrypted indexes on the blockchain-based systems, which aim at secure EHRs sharing with high efficiency. The contribution of this paper includes: (1) a novel blockchain-based EHR access mechanism is provided to support EHRs sharing among hospitals under the control of patients and (2) IPFS is proposed to access large-size EHR files at high speed with the authority of patients.

This paper is organized as follows: Section 2 reviews the related work.  Section 3 illustrates the framework of the secure sharing scheme of EHRs.  Section 4 introduces the experiment and the discussion of the results.  Section 5 discusses the challenges of the proposed scheme and provides some solutions.  Section 6, the last section, shows the conclusion and remarks on future studies.

## 2. Related Work

Blockchain technologies provide new solutions to secure EHRs sharing. As is known in the world, blockchain is a kind of distributed ledger that stores data in blocks and forms a hash chain in chronological order through cryptography and multiparty consensus (see Figure 1) [10, 11]. Based on the features of blockchain [12], scholars seek new ideas for secure data sharing with blockchain technologies [12–16].

In recent years, many scholars have been studying how to use blockchain to securely share EHRs. Yue et al. proposed a blockchain-based access architecture, Healthcare Data Gateway (HDG), which allowed patients to process their own data without invasion of privacy [17]. Azaria et al. proposed a decentralized MedRec that used blockchain to store the hash value of EHR indexes on the blockchain to provide complete data to patients. At the same time, it also used the smart contract to track the transition of some states to improve data privacy protection for patients [8]. Ivan proposed a method based on blockchain to store patient medical records safely. This method allows patients to access and control their own health data. Using existing meaningful usage standards, authorized entities can receive copies of patient data [18]. Xue et al. proposed a blockchain-based medical data sharing model that combined medical institution federation servers (MIF) and auditing federation servers (AFS) with the improved delegate proof of stake mechanism (DPOS) to construct the platform of medical data sharing [19]. Ekblaw et al. proposed a decentralized record management system using blockchain technology to deal with EHRs, which ensured the accuracy of EHRs by using the nontamperable characteristics of blockchain. However, the scheme did not establish policies for data access, which can lead to leakage of medical data [20]. Roehrs et al. integrated distributed EHR with blockchain technology to build a patient-centered medical architecture model. It was argued that the model only integrated the medical data distributed in different medical institutions into view and simply stored the data in the blockchain. Xu et al. proposed a privacy-preserving health chain scheme for large-scale health data management. The work was carried out to provide fine-grained access control for encrypted health data on blockchain. They established two blockchains to ensure that patient data and doctor diagnosis cannot be tampered with [21]. In Mohsin et al.'s study, they argued that even blockchain is used to achieve data integrity and availability, the RSA-based authorization is not unavailable when patients are incapacitated or the encryption keys are forgotten or missed. This problem is ignored in most studies, but it will have a great negative impact on the sharing of medical data. They proposed the integration of finger vein verification with blockchain to solve the problem [22–24].

Due to the limitation of the storage space of the blocks and the low efficiency of data transfer between blocks, the blockchain cannot store the large-size data from the EMR [25, 26]. Esposito et al. also pointed out that although the blockchain contributed much to protecting patients' privacy, data manipulation and sharing inevitably suffered from the low-efficiency puzzle [27]. In recent years, some cloud-based healthcare systems are established to meet the demand for data aggregation. However, the privacy of data in cloud-based frameworks is still under threat [28]. Therefore, many scholars proposed hybrid schemes of blockchain and cloud storage to implement secure and efficient data sharing [29]. In practice, the abstracts of EHRs are published on the blockchain, and the full content of EHRs is encrypted and stored in cloud storage. The indexes of EHRs are embedded in the abstracts. To prevent EHRs from being tampered with, the hash values of EHRs are also stored in the abstracts. For example, Liu et al. proposed a privacy-preserving data sharing scheme (BPDS) based on blockchain technology. In their scheme, medical data are encrypted and stored in the cloud, and the index value of the data in the cloud is written to the blockchain. Visitors can share the data by obtaining the index value and the key. However, in the scheme, visitors are not tracked, and EHRs are not validated whether they are tempered with [30]. Aiming at security and privacy problems in sharing personal medical records, Mei combined blockchain technology and cloud storage technology to design a distributed scheme of security, storage, and sharing of personal medical records. In this scheme, medical records are owned by patients, and data access rights are also owned by patients. Patients can share their medical records with hospitals and medical research institutions. It also has the function to revoke the authority in time to effectively realize the safe storage and effective use of personal medical records [31].

Although, in hybrid models, cloud storage solves the problem of blockchain data storage, some studies point out that the cloud-based storage of various medical institutions is in a centralized storage mode in which the data security itself is still threatened. At the same time, centralized access will also meet the low-efficiency problem of data transmission in the network. In most cases, the proposed hybrid data sharing model still lacks complete robustness and partially meets the high computation load and communication overheads [28]. In addition, most related studies did not concern about the existing/historical data sharing, interaction efficiency, user-friendliness, and integration with existing hospital information systems. In current healthcare settings, these issues should be seriously taken into account for the successful sharing of EHRs.

## 3. The EHRs Sharing Scheme Based on Blockchain and the Interplanetary File System

This paper proposed a new sharing scheme of EHRs based on blockchain and interplanetary file system (IPFS). The proposed scheme has the following features:

1. EHRs are encrypted and distributedly accessed through IPFS, which not only can protect data privacy but also can improve the efficiency of data access.
2. The blockchain saves abstracts of EHRs and access logs. Only authorized users can access medical data in the access control of smart contracts. Once the data are leaked, the authorized organization can trace the malicious entities.
3. With the hash-valued file address of EHR files provided by IPFS, the smart contract ensures the integrity and security of EHR files.
4. The finger vein technology optimizes data authorization, so the sharing of EHRs is guaranteed even if patients are incapacitated or the private keys of patients are forgotten or missed.

Figure 2 shows the framework of the proposed scheme.

In the proposed scheme, the access process of EHRs is divided into five steps as follows:

1. EHRs are generated by doctors or other medical technicians. EHRs refer to abstracts, original documents, and images that should be published to IEFS and BEAS. Since doctors may not have much time to upload medical data in daily work, it may result in delays in patient care. The proposed scheme provides a plug-in installed on doctor workstations to call BEAS.publish (EHR; see Algorithm 1) to upload new EHR data to BEAS and IEFS. Since the public keys of patients are saved in hospital information systems when patients are enrolled at hospitals and the private keys of doctors are read into the memory when they log into workstations, the plug-in can automatically work without interaction with patients and doctors.
2. When doctors want to visit EHRs outside the local hospital information systems, they send requests to BEAS, which forwards requests to patients immediately.
3. When patients get requests, they decrypt the abstracts of requested EHRs with their private keys and re-encrypt EHR file hash addresses with doctors' public keys and return the encrypted addresses to doctors. Concurrently, patients send doctors' IDs to IEFS for access control. To simplify the access process, the time window is usually set as the default value, 24 hours. In most cases, patients have been enrolled at hospitals, so they will deal with the requests in time. If patients are at home or somewhere, the response may be delayed for hours or days. However, the operation of patients is as simple as a click on “agree” button or hyperlink in the messages to their mailboxes or cell phones.
4. When doctors get encrypted addresses, they decrypt them with their private keys and send EHR file access requests to IEFS in the time window. Meanwhile, the visit logs are published to BEAS for auditing. We also strongly propose another plug-in to doctor workstations to run the operations in this step.
5. IEFS checks the doctors' IDs, request time, and file addresses and then returns EHR files to doctors.

### 3.1. The IPFS-Based EHR File System

In the proposed scheme, IPFS is used to develop the EHR file sharing system. As a kind of peer-to-peer distributed file system, IPFS seeks to connect all computing devices with the same system of files. IPFS provides a high-throughput content-addressed block storage model with content-addressed hyperlinks. This forms a generalized MerkleDAG, a data structure upon which one can build versioned file systems, blockchains, and even a Permanent Web. IPFS combines a distributed hash table, an incentivized block exchange, and a self-certifying namespace. Through appropriate redundant backup, IPFS has no single point of failure, and nodes do not need to trust each other [32]. Based on the above technical features, IPFS encrypts, separates, and stores files in a distributed way, which makes the network faster, more secure, and more open. Content-based addressing is an outstanding technical feature of IPFS. With this technology, a unique hash value is generated from the content of the stored file. The hash value is taken as the address access to the file and the validation key against tampering. Therefore, the integration of IPFS with blockchain is a preferred solution to the secure sharing of medical data.

In practice, we use IPFS to store EHR files and publish the invariable and permanent hash addresses of EHR files on the blockchain as validation keys and access indexes. In this study, we suggest that medical institutions participate in the construction of IPFS-based EHR file systems (IEFS). That is, IEFS is a kind of federal system of node servers that belong to each medical institution. Medical institutions that contribute node servers have the rights to request EHRs stored in IEFS. Considering the diversity of EHR data, we suggest that files in each EHR are packed into one file, for example, a zip file, before being submitted to IEFS.

In IEFS, a gateway is responsible for access control. Each request for EHR is validated against the visitor's ID, the time window, and the hash address. If these data do not match those previously submitted by patients (EHR owners), the request will be rejected. The access log is concurrently published to BEAS by the gateway for auditing no matter the request is successful or not.

### 3.2. The Blockchain-Based EHR Abstract System

#### 3.2.1. The Publishing of EHRs

In this study, EHR abstracts are published on blockchain for index and validation. The abstracts are defined in Table 1.

Doctors perform the publish service of BEAS to publish EHR abstracts on blockchain in BEAS. The algorithm of the publish service is shown in Algorithm 1.

In the submit service, the doctor workstation plug-in submits the EHR file to IEFS, gets the hash-valued file address, and encrypts the address by the public key of the patient. Thus, the EHR file address is controlled by the patient himself. When someone wants to visit the EHR file, he has to request the decrypted EHR file address. The doctor workstation plug-in uses the doctor's private key to encrypt the hash value of the main elements of the abstract to generate the signature and sends the abstract data with the signature to BEAS. When BEAS gets the abstract, the smart contract BEAS.*validate_save*() is performed to decrypt the signature with the doctor's public key, produce the new hash value of the abstract, and compare the new hash value with the decrypted signature. If equal, BEAS will publish the EHR abstract on the blockchain.

#### 3.2.2. The Retrieval of EHRs

It is noted that considering the access efficiency of EHRs, elements in EHR abstracts except EHR file addresses are stored in plaintext. Therefore, doctors registered in BEAS are allowed to search EHRs with P_ID, D_ID, H_Name, or Keywords. When getting the required EHR abstracts, doctors send requests for EHR file addresses to BEAS with D_IDs. The requests for HER file addresses are defined in the format shown in Table 2.

If patients accept requests, they will decrypt the EHR file addresses with their private keys (P_SKeys), encrypt them with doctors' public keys (D_PKeys), and return the encrypted addresses to doctors. Meanwhile, they send authorities including D_ID and TimeWindow (usually the default value such as 24 hours) to IEFS. The smart contract *EHR_Retrieve*() of BEAS is responsible for this work. When doctors get encrypted file addresses, they decrypt the addresses with their private keys and send the addresses with their IDs to IEFS. When IEFS gets the requests, it checks doctors' IDs and request time with patients' authority. If the check is passed, IEFS encrypts EHR files with doctors' public keys and returns encrypted EHR files to doctors. The retrieval operations are illustrated in Figure 3.

## 4. Experiment

We conducted an experiment to validate the proposed scheme with a prototype application. We downloaded the installation packages of IPFS [33] and Ethereum [34] from GitHub and installed the IPFS and Ethereum system on CentOS hosts. The environment was composed of 50 computers as blockchain nodes and 50 computers as file hosts. The configuration of each computer is shown in Table 3.

The prototype application consists of an access control module of IEFS and the EHR abstract retrieval and access authorization smart contract on BEAS, which were developed in Java development kits (JDK1.8), Java pairing-based cryptography library (JPBC 2.0.0), Solidity [35], and Tuffle [36]. The experiment system was designed as a typical web application based on hypertext transfer protocol over the secure socket layer protocol (HTTPS), which further implements secure communication.

We prepared an EHR zip file and the abstract data and simulated operations of the doctor (D_ID: ‘0x9249a6bb26d426963E39240853157E5b4498f8E8′') and the patient (P_ID: ‘0x4f98EB5eB7Fe1903c6C53E76c8D82f484443E700') to observe the outputs of important steps.

According to the test report shown in Table 4, the proposed scheme implements the secure sharing of EHRs in an open interconnected environment. In the proposed scheme, EHRs are accessed at a high speed while protected by IPFS and the authority mechanism. Meanwhile, the unique hash-valued file address is published on the blockchain in BEAS. If the EHR file is changed, a new hash address will be generated, which will never be located by BEAS unless published as a new EHR.

We also observed the performance of the prototype system. We took a 350 MB file and simulated the following four major operations of IEFS and BEAS.

1. IEFS: EHR file upload and download
2. BEAS: EHR abstract publish and retrieval

For each configuration with a different number of computers, the operations were repeatedly performed in 10 turns. The median value of execution time was taken as the final result. The results are shown in Figure 4.

We uploaded and downloaded the same file to the Hadoop file system (HDFS) on the computers with the same configuration in Table 2; the median time was nearly over 8,400 milliseconds. Clearly, the more computers in IPFS, the faster the file upload and download, which shows the outstanding performance of IPFS. On the contrary, the more computers in blockchain, the slower the data publishing and retrieval. However, the data retrieval time is within an acceptable range.

## 5. Discussion

While the proposed scheme is undoubtedly a step in the right direction and validated in the prototype experiment, there still exist some problems elaborately dealt with in our study.

### 5.1. The Authorization Is Extended in Some Extreme Situations

Incapacitated patients and key forgetting or missing are extreme situations that make troubles in EHRs sharing. In these situations, we propose two supplementary solutions. One is the private key IC card, with which doctors and patients can easily provide their keys for authorization and data encryption. The other one is the finger vein technology, which has been considered as a novel measure for authorization and data encryption [23–25]. In our study, we extract doctors and patients' finger vein features with a local binary pattern (LBP) algorithm [37, 38] to encrypt their private keys and publish them on a blockchain. The finger vein-based measure is preferred in our opinion since doctors and patients are not subject to carrying private keys storage media and are not afraid of forgetting or missing private keys anymore. For incapacitated patients, this measure is also available unless their finger veins are damaged.

### 5.2. Concerns about the Existing/Historical EHRs Sharing

The sharing of existing or historical HER is not explicitly concerned in the proposed scheme. Although this is not a completely technical problem of the proposed scheme, it does limit the usage of patients' existing/historical EHRs and affect the diagnosis of diseases to some extent. In practice, publishing existing/historical EHRs in IEFS and BEAS requires the cooperation of patients, which can be a time-consuming and laborious task. From the technical perspective, we can develop a server-end daemon to publish the patient's existing/historical EHRs when we get the patients' authority. However, hospitals will worry more about financial and social problems than technology. In our opinion, the government should take actions to finance and help hospitals promote this work since this can be regarded as something of fundamental public healthcare.

For EHRs in hospitals that patients are visiting, doctors can retrieve them from local hospital information systems. This situation is not involved in the proposed scheme.

### 5.3. Integration of the Proposed Scheme with Existing Hospital Information Systems

Hospitals are equipped with hospital information systems, which are regarded as the most complex information systems in the world. It is hard to re-engineer current hospital information systems to implement the proposed EHRs sharing scheme. In this study, the proposed scheme is designed as a typical hybrid platform composed of IEFS and BEAS, which is running alone and exchanges EHRs with hospital information systems. We developed upload and retrieval plug-ins for EHRs exchange (see Figure 5).

Considering doctors are already under time constraints, two plug-ins are implemented as time-efficient and user-friendly as possible. These plug-ins are all installed in doctor workstations. The upload plug-in works as a daemon that monitors the EHR creation event. When a new EHR is created in HIS, the upload plug-in calls BEAS.publish (EHR) to upload the EHR automatically. The operation is transparent to doctors and patients. The retrieval plug-in is run by doctors. Patients use their finger veins to decrypt their private keys and then use the private keys to decrypt EHR file addresses and re-encrypt these addresses with doctors' public keys and send them back to doctors' mailboxes/smartphones or display them on the workstation screen. The retrieval operation only involves one interaction with the patient and two interactions with the doctor.

### 5.4. Who Implements the Proposed Scheme?

The proposed scheme is about secure EHRs sharing among hospitals. As is proposed in Section 3.1, hospitals are encouraged to contribute computing resources to set up the nodes of IEFS (a kind of peer-peer file system) and BEAS (a kind of consortium blockchain). Each hospital will benefit from its contribution in the long run. However, health insurance can also finance the proposed scheme because it may reduce the healthcare compensation with effective EHRs sharing.

## 6. Conclusions

In this paper, the proposed scheme encloses the blockchain technology and the interplanetary file system (IPFS) technology to realize the secure sharing of medical big data at high speed. We developed a prototype system and conducted an experiment with the prototype system. The experimental result shows the following:

1. In the proposed scheme, once the EHR file is published to IEFS, the file is encrypted and read only in IEFS. If the original EHR file is updated, IEFS will generate a new hash-valued file address that is different from the former address stored in BEAS. That means EHR files cannot be tampered with and deleted in the proposed scheme.
2. The original EHR file address submitted to the blockchain is encrypted with the patient's public key. It means that if the visitor does not get the decrypted hash address from the patient, he will never get the EHR file from IEFS. In addition, we add the time window and visitor's identity into the authority, which means that even the visitor has the right EHR file address, he will not be able to access the EHR file either, if his identity and visit time are not accepted by the authority. That is, we realize the controllable access to medical privacy under the control of patients.
3. The IPFS-based file system is much fast than centralized file systems. On the contrary, the retrieval of EHR abstracts is relatively at a lower speed when more computers are added to the blockchain. However, the speed is still within an acceptable range.

In our study, the following practical issues are seriously discussed and partially solved:

1. How to deal with extreme issues such as incapacitated patients and key forgetting or missing. We proposed a finger vein-based solution to these issues.
2. How to use the existing or historical EHR in current hospital systems. In this case, hospitals worry more about financial and social problems than technology. In our opinion, the government should take action to finance and help hospitals promote this work.
3. The effective and efficient interaction with the proposed sharing scheme. We proposed plug-in-based solutions for improving the effectiveness and efficiency of interactions.

It should be noted that (1) the proposed scheme has not been tested in a real production environment. As is known, in the real production environment, the bandwidth, the number of concurrent users, and the configuration of node computers have significant impacts on EHRs sharing. In the future study, we will move the prototype system to Ethereum and IPFS to validate and improve the proposed scheme. (2) In this proposed scheme, we do not consider the impact of policies and laws on the sharing of medical data. In practice, technical mechanisms should be designed in the framework of laws and policies. (3) In this proposed scheme, the economic model has not been considered, even if it is usually taken as an important part of a feasible sharing scheme of data resources. Fortunately, the successful application of digital currency in blockchains will help us design the economic model in the future.

Notwithstanding its limitation, the idea of merging blockchain with interplanetary file system (IPFS) technology is innovative and a step in the right direction. More research is needed to improve EHRs sharing with existing and upcoming hospital information systems to establish an efficient and friendly interoperable environment.[20].

## Figures and Tables

**Figure 1:** The file system of blockchain.

**Figure 2:** The architecture of the proposed scheme of secure EHRs sharing.

**Figure 3:** The flowchart of EHR retrieval operation.

**Figure 4:** The performance of IEFS and BEAS.

**Figure 5:** The integration of the proposed scheme with existing HIS.

**Algorithm 1:** BEAS.publish (EHR).

**Table 1:** The definition of EHR abstracts.

Field name	Description
H_Name	The name of the hospital or other kind of medical institution
Keywords	Keywords of the EHR, which are important search indexes
P_ID	The user ID of the patient
P_PKey	The public key of the patient, which is used to encrypt the EHR file address
D_ID	The user ID of the doctor
D_PKey	The public key of the doctor, which is used to decrypt the signature
Signature	The signature of the doctor, which is used to validate the EHR abstract
H_Address	EHR hash-valued file addresses in IEFS, which are encrypted by P_Pkeys and taken as indexes and validation keys of EHR files

**Table 2:** The definition of EHR file address request.

Parameter	Description	
H_Name	The name of the hospital or other kind of medical institution	At least one
Keywords	Keywords of EHRs	
P_ID	The user ID of the patient	
D_ID	The user ID of the doctor	
D_PKey	The public key of the doctor	Required

**Table 3:** Configuration of computers.

Parameter	Value
CPU	i7-8700K CPU @ 3.20 GHz
Memory	8 GB
Bandwidth	1,000 M
OS	CentOS 7.3
Hard disk	256G

**Table 4:** Report of the prototype system test.

Test scenario	Operation	Observation report	Result
EHR file upload	The doctor submitted the EHR file to IEFS	IEFS successfully returned the hash file address: Qmcm55BkaB9PifiqBwqGDY489z2YXMQEjZYKKY4sz1jnuz	Done

EHR abstract publish	The doctor published the EHR abstract on BEAS	(1) The abstract was successfully published (2) The file address was encrypted with the patient's public key. The new address was ‘4e652982f63d24eb3cbef31f43d999f5a9a3bef3898b44329fab575b702b421a7974ef0f87111b665dac9e124da6de1336d83f2e21c489db30df6042f856a5a6'	Done

Invalid access of EHR file	The visitor tried to visit the EHR file outside the time window	The visit was rejected	Done
	The unauthorized visitor tried to visit the EHR file	The visit was rejected	Done

EHR file address request	The doctor sent the request to BEAS	(1) The doctor's ID and the time window were successfully accepted by IEFS (2) The file address was successfully decrypted by the patient's private key and re-encrypted with the visitor's public key (3) The address was returned to the visitor. The encrypted address was ‘8a2e1348205a9ef5ab1ad22a83c2211063a8127975e5aa32f75d350ce1a3f3bffedd5ddc28fa214c52926ac679e7ab7462515dfa9708e437db3b5a1723d69556'	Done

EHR file download	The doctor sent the request to IEFS	(1) The file address was decrypted with the doctor's private key to the original value ‘Qmcm55BkaB9PifiqBwqGDY489z2YXMQEjZYKKY4sz1jnuz' (2) The doctor's ID and the visit time were accepted (3) The file was output by IPFS and encrypted with the doctor's public key (4) The visit log was published to BEAS for auditing (5) The doctor got the file and decrypted it to the original file	Done

## Data Availability

The data about the experiment used to support the findings of this study are available from the corresponding author upon request.

## References

[1] Raham M. S., Khalil I., Arachchige P. C. M. A novel architecture for tamper proof electronic health record management system using blockchain wrapper.

[2] Xue T., Fu Q., Wang C., Wang X. (2017). A medical data sharing model via blockchain. *Acta Automatica Sinica*.

[3] Jensen P. B., Jensen L. J., Brunak S. (2012). Mining electronic health records: towards better research applications and clinical care. *Nature Reviews Genetics*.

[4] Information Center of Ministry of Industry and Information Technology of the People’s Republic of China (May 20th, 2018). The 2018 white paper on China’s blockchain industry. http://www.miit.gov.cn/n1146290/n1146402/n1146445/c6180238/part/6180297.pdf.

[5] Al Omar A., Bhuiyan M. Z. A., Basu A. (2019). Privacy-friendly platform for healthcare data incloud based on blockchain environment. *Future Generation Computer Systems*.

[6] AbuKhousa E., Mohamed N., Al Jaroodi J. (2012). E-health cloud: opportunities and challenges. *Future Internet*.

[7] Hölbl M., Kompara M., Kamišali´c A., Zlatolas L. N. (2018). A systematic review of the use of blockchain in healthcare. *Symmetry*.

[8] Azaria A., Ekblaw A., Vieira T. Medrec: using blockchain for medical data access andpermission management.

[9] Hoerbst A., Ammenwerth E., Hoerbst A. (2010). Electronic health records. A systematic review on quality requirements. *Methods of Information in Medicine*.

[10] S N., Bitcoin (2019). A peer-to-peer electronic cash system. https://bitcoin.org/bitcoin.pdf.

[11] Shao Q., Jin C., Zhang Z. (2018). Blockchian: architecture and research progress. *Chinese Jorunal of Computers*.

[12] Yuan Y., Wang F. (2016). Blockchian: the state of the art and futrue trends. *Acta Automatica Sinica*.

[13] Zheng Z., Xie S., Dai H. N., Chen X., Wang H. (2018). Blockchain challenges and opportunities: a survey. *International Journal of Web and Grid Services*.

[14] Zheng Z., Xie S., Dai H. An overview of blockchain technology: architecture, consensus, and future trends.

[15] McGhin T., Choo K.-K. R., Liu C. Z., He D. (2019). Blockchain in healthcare applications: research challenges and opportunities. *Journal of Network and Computer Applications*.

[16] Loizou C., Karastoyanova D., Schizas C. Measuring the impact of blockchain on healthcare applications.

[17] Yue X., Wang H., Jin D., Li M., Jiang W. (2016). Healthcare data gate-ways: found healthcare intelligence on blockchain with novel privacy risk control. *Journal of Medical Systems*.

[18] Ivan D. (2016). Moving toward a Blockchain-Based Method for the Secure Storage of Patient Records. https://www.healthit.gov/sites/default/files/9-16-drew_ivan_20160804_blockchain_for_healthcare_final.pdf.

[19] Xue T., Fu C., Wang C., Wang X. (2017). A medical data sharing model via blockchain. *Acta Automatica Sinica*.

[20] Ekblaw A., Azaria A., Halamka J. D. (2016). A case study for blockchain in healthcare: “MedRec” prototype for electronic health records and medical research data. *Proceedings of IEEE open ＆ big data conference*.

[21] Xu J., Xue K., Li S. (2019). Healthchain: a blockchain-based privacy preserving scheme for large-scale health data. *IEEE Internet of Things Journal*.

[22] Mohsin A. H., Zaidan A. A., Zaidan B. B. (2019). Blockchain authentication of network applications: taxonomy, classification, capabilities, open challenges, motivations, recommendations and future directions. *Computer Standards & Interfaces*.

[23] Mohsin A. H., Zaidan A. A., Zaidan B. B. (2019). Based blockchain-PSO-AES techniques in finger vein biometrics: a novel verification secure framework for patient authentication. *Computer Standards & Interfaces*.

[24] Mohsin A. H., Zaidan A. A., Zaidan B. B. (2021). PSO-Blockchain-based image steganography: towards a new method to secure updating and sharing COVID-19 data in decentralised hospitals intelligence architecture. *Multimedia Tools and Applications*.

[25] Zhai S., Wang Y., Cheng S. (2020). Research on the application of blockchain technology in the sharing of electronic medical records. *Journal of Xidian University*.

[26] Roehrs A., Goldim J. R., Schmidt D. C. (2019). Analyzing the performance of a blockchain-based personal health record implementation. *Journal of Biomedical Informatics*.

[27] Esposito C., De Santis A., Tortora G., Chang H., Choo K.-K. R. (2018). Blockchain: a panacea for healthcare cloud-based data security and privacy? blockchain: apanacea for healthcare cloud-based data security and privacy?. *IEEE Cloud Computing*.

[28] Shanthapriya R., Vaithianathan V. (2020). Block-healthnet: security based healthcare system using blockchain technology. *Security Journal*.

[29] Park J., Park J. (2017). Blockchain security in cloud computing: use cases, challenges, and solutions. *Symmetry*.

[30] Liu J., Li X., Ye L. BPDS: a blockchain based privacy-preserving data sharing for electronic medical records.

[31] Mei Y. (2017). The utilizing blockchain-based method of the secure storage of medical records. *Journal of Jiangxi Normal University (Natural Science)*.

[32] Juan B. (2014). IPFS-content Addressed, Versioned, P2P File System. https://github.com/ipfs/ipfs/blob/master/papers/ipfs-cap2pfs/ipfs-p2p-file-system.pdf%20(or%20https://arxiv.org/pdf/1407.3561v1.pdf.

[33] (2021). IPFS: A Peer-To-Peer Hypermedia Protocol. https://github.com/ipfs.

[34] (2021). Go-ethereum. https://github.com/ethereum/go-ethereum.

[35] (2021). Solidity. https://github.com/ethereum/solidity.

[36] (2021). Sweet Tools for Smart Contracts. https://www.trufflesuite.com.

[37] You L., Wang J., Yan B. (2016). A secure finger vein recognition algorithm based on MB-GLBP and Logistic mapping. *Journal of information hiding and multimedia signal processing*.

[38] Ojala T., Pietikainen M., Maenpaa T. (2002). Multiresolution gray-scale and rotation invariant texture classification with local binary patterns. *IEEE Transactions on Pattern Analysis and Machine Intelligence*.

